# Circular RNA Hsa_circ_0006766 targets microRNA miR-4739 to regulate osteogenic differentiation of human bone marrow mesenchymal stem cells

**DOI:** 10.1080/21655979.2021.1967712

**Published:** 2021-09-15

**Authors:** Zhaodi Guo, Manlin Xie, Yanfang Zou, Qianxin Liang, Fubin Liu, Jing Su, Zhiliang He, Xiuping Cai, Zhixiang Chen, Qing Zhao, Kewei Zhao

**Affiliations:** a The Clinical laboratory, The Third Affiliated Hospital of Guangzhou University of Chinese Medicine, Guangzhou, Guangdong, China; b The Third Clinical Medical College, Guangzhou University of Chinese Medicine, Guangzhou, Guangdong, China

**Keywords:** circRNA, miRNA, hBM-MSCs, osteogenesis

## Abstract

Circular RNAs (circRNAs) are emerging as important regulators in bone metabolism, which is mediated by microRNA (miRNA) sponges. However, it is not clear how circRNA regulates osteogenic differentiation of human bone marrow mesenchymal stem cells (hBM-MSCs).Therefore, based on the previous circRNA chip results, hsa_circ_0006766, which is differentially expressed in the osteogenic differentiation of hBM-MSCs, was screened out, and bioinformatics analysis was performed to predict potential target miRNAs. During osteogenic differentiation of hBM-MSCs, hsa_circ_0006766 and its target miRNAs (miR-4739, miR-619-5p, miR-5787, miR-7851-3p, and miR-3192-5p) were detected by quantitative Real Time-PCR (qRT-PCR). Target gene prediction for the differentially expressed target miRNAs was performed, and target genes were validated by dual-luciferase reporter gene assay and qRT-PCR. It is shown that hsa_circ_0006766 was up-regulated and miR-4739 was down-regulated during osteogenic differentiation of hBM-MSCs.Moreover, the target gene Notch2 was predicted to be highly expressed during osteogenic differentiation. And dual-luciferase assay proved that Notch2 was the gene targeting to miR-4739. Taken together, our finding confirmed that hsa_circ_0006766 may act as a major regulatory part in osteogenic differentiation of hBM-MSCs via an hsa_circ_0006766–miR-4739–Notch2 regulatory axis. Accordingly, hsa_circ_0006766 may affect the development of osteoporosis and may thus become a therapeutic target.

## Introduction

Osteoporosis (OP) is the most common metabolic bone-related disease in which bone density and bone quality are decreased, bone microstructure is destroyed, and bone fragility is increased, thereby prone to fracture[1]. One of the mechanisms of OP is the imbalance of differentiation of mesenchymal stem cells from bone marrow (BM-MSCs) into osteoblasts and adipocytes, resulting in a decrease of osteoblasts and an increase of adipocytes[2].

circRNA exhibits a circular structure, which cannot be degraded by RNA exonucleases, and has strong stability [3–5], can serve as a microRNA (miRNA) sponge to relieve the effect of inhibition of miRNA on its target gene and enhance its expression [6–8]. Previous reports have shown that circular RNA (circRNA) has vital regulatory functions in all kinds of stem cells’ osteogenic differentiation. For example, circRNA_33287 regulates osteogenic differentiation of maxillary sinus membrane stem cells through the circRNA_33287/miR-214-3p/Runx3 axis[9]. Through negatively regulating microRNA-7, CircRNA CDR1as can regulate osteogenic differentiation process of periodontal ligament stem cells, specifically, firstly, CDR1as/microRNA-7 partially via regulating GDF5, then CDR1as/GDF5 partly by enhanced p38 MAPK phosphorylation[10].Furthermore, circRNA can regulate bone metabolism via the circRNA-miRNA-mRNA network and influence the occurrence and the development of diseases associated with bone metabolism [11–14]. Recent researches have confirmed that circRNA may act as a main regulatory part in the differentiation and proliferation of BM-MSCs [15,16]. But so far, the specific role of circRNA in the osteogenic differentiation of human BM-MSCs (hBM-MSCs) is not yet clear. Our previous circRNA microarray results found that hsa_circ_0006766 is up-regulated in peripheral blood mononuclear cells derived from patients with postmenopausal osteoporosis[17], but the specific mechanism in osteogenic differentiation of hBM-MSCs is not yet clear, and it is worthy of our in-depth discussion.

We aimed to confirm the role of hsa_circ_0006766 in the process of osteogenic differentiation of hBM-MSCs in this study. We assume that hsa_circ_0006766 may promote the osteogenic differentiation of hBM-MSCs through the hsa_circ_0006766–miR-4739–Notch2 axis, and therefore may become an effective biomarker for the prognosis and diagnosis of osteoporosis.

## Methods

### Cell culture

hBM-MSCs (Saliai, Guangzhou, China) were cultured in human bone marrow mesenchymal stem cell-specific medium (Cyagen, Santa Clara, CA, USA), and HEK-293 T cells (Sun Yat-sen University, Guangzhou, China) were cultured in Dulbecco’s Modified Eagle’s Medium-high glucose (Gibco, Grand Island, NY, USA), which contains 10% FBS,1% 100× Penicillin-Streptomycin Solution (Gibco) in an incubator.

### Osteogenic differentiation of hBM-MSCs

hBM-MSCs cultured to passage 5 were inoculated into 6-well plate with 2 × 10^5^ per well and further cultured in a 37°C constant temperature. When grown to almost 80%, the medium was changed to mesenchymal stem cell osteogenic differentiation solution (Caygen), and then changed once every 2–3 days.

### Alizarin red staining

Cells that underwent osteogenic differentiation for 14 days were stained with Alizarin Red. After the cells were fixed with 4% paraformaldehyde for 30 min, washed with PBS. Added with 1 ml of Alizarin Red S dye solution, stood at room temperature for 3–5 min. Using PBS to wash cells one more time, and mineralization was subsequently observed and imaged using an inverted microscope.

### Bioinformatics analysis

TargetScan 7.2 and miRanda miRNA target gene prediction software were used to predict miRNA response elements (MREs) within hsa_circ_0006766. After target gene prediction, the miRNAs were classified by functional enrichment analysis based on the Gene Ontology (GO) database. The accession numbers of the target genes were used as clues for tracking. GO annotations were obtained from the UCSC Genome Browser. Next, miRNAs with significant differences in expression levels were categorized and classified. Kyoto Encyclopedia of Genes and Genomes (KEGG) mapping was performed basing on GO annotations, and statistical methods such as hypergeometric distribution tests were used to determine significantly enriched biological signaling or metabolic pathways. Through pathway analysis of differentially expressed genes, we identified enriched pathways.

### RNA extraction and quantitative Real Time-PCR (qRT-PCR) analysis

The gene sequences were downloaded from the NCBI or miRbase databases; the associated primer sequences are shown in Table 1. hBM-MSCs were induced to differentiate for 0, 1, 3, and 7 days, after which total RNA was extracted and purified per the instructions of the QIAzol Lysis Reagent (Qiagen, Hilden, Germany). After the total RNA quality test was qualified, RNA was transcribed into cDNA per the instructions of the Takara reverse transcription kit (Kusatsu, Japan). The cDNA template obtained from reverse transcription was added to the detection system per the instructions of the Takara real-time fluorescence quantitative PCR kit, and the reaction was performed using the Qiagen real-time fluorescence quantitative PCR analyzer. *U6* and Human β-actin were selected as house-keeping genes for miRNAs and circRNAs or mRNAs, respectively. Each sample was run in triplicate. Relative quantitation was performed by comparing threshold cycle (CT) values. Finally, differences in target gene expression were analyzed using the 2^−ΔΔCT^ relative quantification.

**Table 1.** Primers for real time PCR

Gene	5′-3′ (Forward)	3′-5′ (Reverse)
β-actin	TGACGTGGACATCCGCAAAG	CTGGAAGGTGGACAGCGAGG
hsa_circ_0006766	CCCTATCCCT TTTCCATATC	CTAACTTACC CCTGTAATGG
ALP	CCAACCTGAGCTGCCTTTCTCA	GCTTCTCCCCTCGTTGCCA
RUNX2	GACCGTGGTTACCGTCATGGC	ACTTGGTTTTTCATAACAGCAGA
Notch2	CAGGCACTCGGGGTATGAAA	ATGCCCTGGATGGAAAATGGA
ZFP36L1	CCCGACCTTGGACAACTCAA	CTGCAGACCCTGGCTTAGTC
Wnt1	ACCTCTTCGGCAAGATCGTC	GTTTCTCGACAGCCTCGGTT
U6	CTCGCTTCGGCAGCACA	
hsa-miR-4739	AAGGGAGGAGGAGCGGAGGGGCCCT	
hsa-miR-619-5p	GCTGGGATTACAGGCATGAGCC	
hsa-miR-5787	GGGCTGGGGCGCGGGGAGGT	
hsa-miR-7851-3p	TACCTGGGAGACTTGAGGTTGGA	
hsa-miR-3192-5p	TCTGGGAGGTTGTAGCAGTGGAA	

### Dual luciferase reporter gene assay

HEK293T cells were co-transfected with miR-4739 mimic/negative control and Notch2, Wnt1, or ZFP36L1 wild-type or mutant 3ʹ-untranslated region (UTR) reporter plasmid. Using Dual Luciferase Reporter Gene Assay Kit (Beyotime, Shanghai, China) to measure the firefly and Renilla luciferase values based on the provided manual after 48 h of transfection. All assays were repeated no less than thrice.

### Statistical analysis

With the use of GraphPad Prism v7.0 statistical software, one-way analysis of variance was employed for multiple group testing, and the Mann–Whitney test for non-parametric was used to analyze the differences between groups. *P* value of less than 0.05 was regarded as significant.

## Results

In this study, we inspected the changes of hsa_circ_0006766 during the osteogenic differentiation of hBM-MSCs by inducing the osteogenic differentiation of it. Through bioinformatics, qRT-PCR and dual luciferase, we proved that hsa_circ_0006766 may promote the osteogenic differentiation of hBM-MSCs via hsa_circ_0006766–miR-4739 -Notch2 axis .

### Osteogenic culture of hBM-MSCs

Firstly, in order to confirm the successful induction of hBM-MSCs, Alizarin Red staining was performed. Cell aggregates were observed on day 7 of osteogenic differentiation of hBM-MSCs. Brown calcified nodules were observed on day 14, and Alizarin Red staining revealed red calcified nodules, indicating a positive staining result (Figure 1a). Compared with those at day 0, the expression levels of mRNAs, such as ALP and RUNX2, associated with osteogenic differentiation were significantly higher at day 7 after osteogenic differentiation (P < 0.01,Figure 1b).

**Figure 1.** Differentiation of hBM-MSCs into osteoblasts. (a) Alizarin Red staining of hBM-MSCs shows a large number of calcified nodules in 14 days. (b) Relative mRNA expression of *ALP* and *RUNX2* during osteogenic differentiation of hBM-MSCs determined by qRT-PCR. *ns*, not significant relative to D0 group, *P* > 0.05; *P < 0.05; **P < 0.01

### Expression of hsa_circ_0006766 during osteogenic differentiation of hBM-MSCs and construction of a circRNA–miRNA–mRNA network

In order to confirm that hsa_circ_0006766 is up-regulated during the osteogenic differentiation of hBM-MSCs, we used qRT-PCR to verify and constructed a circRNA-miRNA-mRNA network to find the downstream target genes of hsa_circ_0006766. qRT-PCR results showed that during 7 days of induction of osteogenic differentiation, hsa_circ_0006766 expression in hBM-MSCs significantly increased with time compared with that on day 0 (*P* < 0.01, Figure 2a). Hsa_circ_0006766 was predicted to interact with five miRNAs (hsa-miR-4739, hsa-miR-619-5p, hsa-miR-5787, hsa-miR-7851-3p, and hsa-miR-3192-5p) (Figure 2b). The prediction system was then used for identifying target genes of these miRNAs and a network of circRNA-miRNA-mRNA interaction was plotted using Cytoscape (Figure 2b).

**Figure 2.** Construction of circRNA–miRNA–mRNA network and expression of hsa_circ_0006766 during osteogenic differentiation of hBM-MSCs. (a) Relative expression of hsa_circ_0006766 during osteoblastic differentiation of hBM-MSCs as determined by qRT-PCR analysis. *ns*, not significant relative to D0 group, *P* > 0.05; * *P* < 0.05; ** *P* < 0.01. (b) The network of circRNA–miRNA–mRNA consisting of hsa_circ_0006766(green node), target miRNAs (yellow squares) and their target mRNAs(blue nodes), in which the bone metabolism related target mRNAs is marked with red

### Hsa_circ_0006766 functional enrichment analysis

The functional enrichment and pathway of hsa_circ_0006766 regulating the osteogenic differentiation of hBM-MSCs was further analyzed by bioinformatics. GO analysis showed that the target genes regulated by the five miRNAs related with hsa_circ_0006766 were primarily enriched in biological processes (BP) (Figure 3a), particularly the regulation of signaling and regulation of cell communication (Figure 3b). The possible signal pathways of hsa_circ_0006766 are predicted by KEGG Pathway analysis (Figure 3c). Of these, the MAPK signaling pathway is closely associated with bone metabolism (Figure 3d).

**Figure 3.** Functional and pathway enrichment analysis of hsa_circ_0006766. (a) Results of GO analysis. (b) Top 10 GO terms (biological processes) determined by GO analysis according to the enrichment score. (c) Top 10 pathways determined by KEGG analysis according to the enrichment score. (d) Map of hsa_circ_0006766-mediated MAPK signaling pathway

### Expression of miRNAs targeted by hsa_circ_0006766 during osteogenic differentiation of hBM-MSCs

It was verified by qRT-PCR whether miR-4739 is the target miRNA of hsa_circ_0006766, and the target genes related to the regulation of bone metabolism by miR-4739 were found through bioinformatics analysis. qRT-PCR analysis showed that miR-4739 was the only target miRNA significantly downregulated within 7 days after induction of osteogenic differentiation, compared with levels in uninduced hBM-MSCs (*P* < 0.05, Figure 4a). *Notch2, ZFP36L1*, and *Wnt1*, which are associated with bone metabolism and were predicted to be target genes of miR-4739 (Figure 2b), were significantly upregulated (*P* < 0.05; Figure 4f, Figure 4g, and Figure 4h, respectively). CircRNA profile data demonstrated four binding sites of the coding sequence for hsa_circ_0006766 in miRNA-4739 (Figure 5a).

**Figure 4.** Relative expression of the predicted target miRNAs of hsa_circ_0006766 determined by qRT-PCR. (a–e) Expression of the five predicted MREs of hsa_circ_0006766. (f–h) Expression of the predicted target genes of miR-4739 related to bone metabolism. *ns*, not significant relative to D0 group, *P* > 0.05; *P < 0.05; **P < 0.01; ***P < 0.001; ****P < 0.0001

**Figure 5.** Dual luciferase reporter detection of target genes of miR-4739. (a)Detailed annotation map of hsa_circ_0006766 with miR-4739. Only the binding sites of the coding sequence in hsa_circ_0006766 are shown.(b) Predicted binding sites of miR-4739 in *Notch2, ZFP36L1*, and *Wnt1* determined by TargetScan. Relative luciferase activities in cells overexpressing miR-4739 with wild-type or mutated miR-4739 binding sites in (c) *Notch2*, (d) *ZFP36L1*, and (e) *Wnt1. ns*, not significant, *P* > 0.05; ** *P* < 0.01; ****P < 0.0001

### Dual-luciferase reporter gene assay

In order to confirm that Notch2 is a downstream target gene of miR-4739, a dual luciferase reporter analysis was performed. TargetScan revealed the 3ʹ-UTR binding site of the miR-4739 target genes Notch2, ZFP36L1, and Wnt1 (Figure 5b). Based on the dual-luciferase reporter gene analysis, the miR-4739 mimic significantly suppressed the expression of the target gene Notch2 after transfection of the wild-type plasmid related to the negative control (P < 0.05, Figure 5c). Additionally, Notch2 expression was restored after mutation of the binding site (P < 0.05, Figure 5c). Conversely, the expression of the target genes ZFP36L1 and Wnt1 were not inhibited by the transfection of miR-4739 mimic in wild-type plasmid (Figure 5d and Figure 5e). These results indicated that among the predicted genes, Notch2, but not ZFP36L1 or Wnt1, is a target gene of miR-4739.

## Discussion

circRNA plays a huge role in many diseases [18,19]. It not only primarily acts as an miRNA sponge, but can also regulate gene transcription, interplay of RNA-binding proteins, and participate in protein translation [20,21]. Previous studies have demonstrated that differential expression of circRNA hsa_circ_0001275 may become a potential new diagnostic biomarker in patients with postmenopausal OP[17], while circRUNX2 can bind to miR-203 and enhance the expression of RUNX2, thereby preventing OP[22]. It is reported that a great deal of miRNAs are participated in bone formation[23]. But in fact, few studies have paid attention to the relevance and function of circRNAs in osteogenic differentiation of hBM-MSCs.

We previously observed significant differential expression of hsa_circ_0006766 in patients with postmenopausal OP based on circRNA chip results. During the induction of osteogenic differentiation of hBM-MSCs, we discovered that hsa_circ_0006766 significantly increased. Therefore, we speculated that hsa_circ_0006766 is highly correlated with osteogenic differentiation of hBM-MSCs. Only one target miRNA (MiR-4739) which was discovered to be significantly downregulated in osteogenic differentiation of hBM-MSCs. MiR-4739 was reported to be closely associated with bone metabolism and is involved in the process of regulating the osteogenic differentiation of hBM-MSCs[24]. These results suggest that *Notch2* is a target gene of miR-4739.

Studies have indicated that circRNA can affect the development of diseases by regulating signal transduction pathways [25,26]. Through KEGG pathway analysis, we found that hsa_circ_0006766 mediates MAPK signaling, which is involved in bone metabolism, and that Notch2 regulates the MAPK signaling pathway. In addition, ERK1/2, p38-MAPK, and JNK pathways within the MAPK signaling pathway are closely associated with osteogenesis of bone marrow mesenchymal stem cells and treatment of OP [27–30]. Inducing osteogenic differentiation of mesenchymal stem cells from bone marrow (BM-MSCs), the phosphorylation of ERK and p38 plays a crucial effect in regulating osteogenic differentiation and promoting bone formation [31,32]. Activation of ERK signaling in the MAPK pathway promotes the stimulation of osteogenic differentiation of BM-MSCs by BMP2/7 growth factors[33]. p38 and ERK1/2 have significant functions in BMP9-induced osteogenic differentiation of BM-MSCs by influencing the canonical Smad signaling pathway[34]. BMP9-induced BMP9 activity and BMP/Smad signaling in BM-MSCs are enhanced by Notch signaling, thus inducing osteogenic differentiation of BM-MSCs[35]. Therefore, based on the results of our study and related reports, we suggest that hsa_circ_0006766 promotes osteogenic differentiation of hBM-MSCs through an hsa_circ_0006766–miR-4739–Notch2 axis, specifically by enhancing the expression of Notch2 and regulating the MAPK signaling pathway.

The study had some shortcomings: the functions and mechanisms of hsa_circ_0006766 and the osteogenic differentiation of miR-4739 in hBM-MSCs were not determined by their overexpression or silencing. In addition, the expression of MAPK signaling pathway-related genes was not confirmed by qRT-PCR or western blot. Therefore, the specific mechanism of hsa_circ_0006766 in osteogenic differentiation of hBM-MSCs requires further investigation.

## Conclusion

In summary, we hypothesize that hsa_circ_0006766 regulates the MAPK signaling pathway through a hsa_circ_0006766–miR-4739–Notch2 axis to promote osteogenic differentiation of hBM-MSCs and osteogenesis, which may prevent OP. Overexpression of hsa_circ_0006766 or inhibition of miR-4739 can promote osteogenesis, suggesting new targets for the diagnosis, treatment, and prevention of OP.

## Highlight

1, Hsa_circ_0006766 promotes osteogenic differentiation of hBM-MSCs.

2, Hsa_circ_0006766 directly target miR-4739 and downregulated miR-4739 expression.

3, Notch2 is the target gene of miR-4739.

4, Hsa_circ_0006766 can regulate the MAPK signaling pathway to promote the osteogenic differentiation of hBM-MSCs through the hsa-circ-0006766/miR-4739/Notch2 regulatory axis.

## References

[1] Chinese society of bone and mineral research.Guidelines for diagnosis and treatment of primary osteoporosis(2017). J Chinese J Osteoporosis Bone Mineral Salt. 2017; 10(5):413–443.

[2] Zhanpeng L, Yuanzheng M. Osteoporosis and mesenchymal stem cells[J]. Chinese J Multiple Organ Dis Elderly. 2011;5:388–392.

[3] Li Y, Zheng F, Xiao X, et al. CircHIPK3 sponges miR-558 to suppress heparanase expression in bladder cancer cells[J]. EMBO Rep. 2017;18(9):1646–1659.2879420210.15252/embr.201643581PMC5579470

[4] Hollensen AK, Thomsen R, Bak RO, et al. Improved microRNA suppression by WPRE-linked tough decoy microRNA sponges[J]. RNA. 2017;23(8):1247–1258.2848738110.1261/rna.061192.117PMC5513069

[5] Kang S, Park S, Yoon S, et al. Machine learning-based identification of endogenous cellular microRNA sponges against viral microRNAs[J]. Methods. 2017;129:33–40.2832304010.1016/j.ymeth.2017.03.017

[6] Zheng Q, Bao C, Guo W, et al. Circular RNA profiling reveals an abundant circHIPK3 that regulates cell growth by sponging multiple miRNAs[J]. Nat Commun. 2016;7(1):11215–11227.2705039210.1038/ncomms11215PMC4823868

[7] Tay FC, Lim JK, Zhu H, et al. Using artificial microRNA sponges to achieve microRNA loss-of-function in cancer cells[J]. Adv Drug Deliv Rev. 2015;81:117–127.2485953410.1016/j.addr.2014.05.010

[8] Kulcheski FR, Christoff AP, Margis R. Circular RNAs are miRNA sponges and can be used as a new class of biomarker[J]. J Biotechnol. 2016;238:42–51.2767169810.1016/j.jbiotec.2016.09.011

[9] Penga W, Zhua S, Chen J, et al. Hsa_circRNA_33287 promotes the osteogenic differentiation of maxillary sinus membrane stem cells via miR-214-3p/Runx3[J]. Biomed Pharmacother. 2019;109:1709–1717.3055142510.1016/j.biopha.2018.10.159

[10] Xiaobei L, Zheng Y, Zheng Y, et al. Circular RNA CDR1as regulates osteoblastic differentiation of periodontal ligament stem cells via the miR-7/GDF5/SMAD and p38 MAPK signaling pathway[J].Stem. Stem Cell Research & Therapy. 2018;9(1):232–246.3017061710.1186/s13287-018-0976-0PMC6119336

[11] Wu Z, Shi W, Jiang C. Overexpressing circular RNA hsa_circ_0002052 impairs osteosarcoma progression via inhibiting Wnt/β-catenin pathway by regulating miR-1205/APC2 axis[J]. Biochemical and Biophysical Research Communications. 2018;502(4):465–471.2985216810.1016/j.bbrc.2018.05.184

[12] Deng N, Li L, Gao J, et al. Hsa_circ_0009910 promotes carcinogenesis by promoting the expression of miR-449a target IL6R in osteosarcoma[J]. Biochem Biophys Res Commun. 2018;495(1):189–196.2911753910.1016/j.bbrc.2017.11.028

[13] Zhang H, Wang G, Ding C, et al. Increased circular RNA UBAP2 acts as a sponge of miR-143 to promote osteosarcoma progression[J]. Oncotarget. 2017;8(37):61687–61697.2897789610.18632/oncotarget.18671PMC5617456

[14] Li L, Guo L, Yin G, et al. Upregulation of circular RNA circ_0001721 predicts unfavorable prognosis in osteosarcoma and facilitates cell progression via sponging miR-569 and miR-599[J]. Biomed Pharmacother. 2019;109:226–232.3039608010.1016/j.biopha.2018.10.072

[15] Xiaoyun L, Peng B, Zhu X, et al. Changes in related circular RNAs following ERβ knockdown and the relationship to rBMSC osteogenesis[J]. Biochem Biophys Res Commun. 2017;493(1):100–107.2891941410.1016/j.bbrc.2017.09.068

[16] Zhang M, Jia L, Zheng Y. circRNA expression profiles in human bone marrow stem cells undergoing osteoblast differentiation[J]. Stem Cell Rev Rep. 2019;15(1):126–138.3004699110.1007/s12015-018-9841-x

[17] Zhao K, Zhao Q, Guo Z, et al. Hsa_Circ_0001275: a potential novel diagnostic biomarker for postmenopausal osteoporosis [J]. Cell Physiol Biochem. 2018;46(6):2508–2516.2974250310.1159/000489657

[18] Shen S, Wu Y, Chen J, et al. CircSERPINE2 protects against osteoarthritis by targeting miR-1271 and ETS-related gene[J]. Ann Rheum Dis. 2019;1–11. DOI:10.1136/annrheumdis-2018-214786.30923232PMC6579553

[19] Zhao ZJ, Shen J. Circular RNA participates in the carcinogenesis and the malignant behavior of cancer. RNA Biol. 2017;14(5):514–521.2664977410.1080/15476286.2015.1122162PMC5449088

[20] Huang S, Yang B, Chen BJ, et al. The emerging role of circular RNAs in transcriptome regulation[J]. Genomics. 2017;109(5–6):401–407.2865564110.1016/j.ygeno.2017.06.005

[21] Greene J, Am B, Brady L, et al. Circular RNAs: biogenesis, Function and Role in Human Diseases[J]. Front Mol Biosci. 2017;4:38–48.2863458310.3389/fmolb.2017.00038PMC5459888

[22] Yin Q, Wang J, Fu Q, et al. CircRUNX2 through has-miR-203 regulates RUNX2 to prevent osteoporosis[J]. J Cell Mol Med. 2018;22(12):6112–6121.3032471810.1111/jcmm.13888PMC6237596

[23] Sriram M, Sainitya R, Kalyanaraman V, et al. Biomaterials mediated microRNA delivery for bone tissue engineering[J].Int. International Journal of Biological Macromolecules. 2015;74:404–412.2554306210.1016/j.ijbiomac.2014.12.034

[24] Elsafadi M, Manikandan M, Alajez NM, et al. MicroRNA-4739 regulates osteogenic and adipocytic differentiation of immortalized human bone marrow stromal cells via targeting LRP3[J]. Stem Cell Res. 2017;20:94–104.2834048710.1016/j.scr.2017.03.001

[25] Li F, Zhang L, Li W, et al. Circular RNA ITCH has inhibitory effect on ESCC by suppressing the Wnt/β-catenin pathway[J]. Oncotarget. 2015;6(8):6001–6013.2574938910.18632/oncotarget.3469PMC4467417

[26] Yao Y, Hua Q, Zhou Y. CircRNA has_circ_0006427 suppresses the progression of lung adenocarcinoma by regulating miR-6783–3p/DKK1 axis and inactivating Wnt/β-catenin signaling pathway. Biochem Biophys Res Commun. 2019;508(1):37–45.3047057010.1016/j.bbrc.2018.11.079

[27] Kim HK, Kim M-G, Leem KH. Osteogenic activity of collagen peptide via ERK/MAPK pathway mediated boosting of collagen synthesis and its therapeutic efficacy in osteoporotic bone by back-scattered electron imaging and microarchitecture analysis. Molecules. 2013;18(12):15474–15489.2435200810.3390/molecules181215474PMC6269989

[28] Yang X, Yang Y, Zhou S, et al. Puerarin stimulates osteogenic differentiation and bone formation through the ERK1/2 and p38-MAPK signaling pathways[J]. Curr Mol Med. 2018;17(7):488–496.2925635210.2174/1566524018666171219101142

[29] Zhu D, Deng X, Han X-F, et al. Wedelolactone enhances osteoblastogenesis through ERK- and JNK-mediated BMP2 expression and Smad/1/5/8 Phosphorylation. Molecules. 2018;23(3):561.10.3390/molecules23030561PMC601795929498687

[30] Guo Y, Lianhua L, Gao J, et al. miR-214 suppresses the osteogenic differentiation of bone marrow-derived mesenchymal stem cells and these effects are mediated through the inhibition of the JNK and p38 pathways. Int J Mol Med. 2017;39(1):71–80.2795939410.3892/ijmm.2016.2826PMC5179177

[31] Nan H, Feng C, Jiang Y, et al. Regulative effect of Mir-205 on osteogenic differentiation of bone mesenchymal stem cells (BMSCs): possible role of SATB2/Runx2 and ERK/MAPK pathway[J]. Int J Mol Sci. 2015;16(12):10491–10506.2596195510.3390/ijms160510491PMC4463658

[32] Jaiswal RK, Jaiswal N, Bruder SP, et al. Adult human mesenchymal stem cell differentiation to the osteogenic or adipogenic lineage is regulated by mitogen-activated protein kinase[J]. J Biol Chem. 2000;275(13):9645–9652.1073411610.1074/jbc.275.13.9645

[33] Miao C, Qin D, Cao P, et al. BMP2/7 heterodimer enhances osteogenic differentiation of rat BMSCs via ERK signaling compared with respective homodimers[J]. J Cell Biochem. 2019;120(5):8754–8763.10.1002/jcb.2816230485526

[34] Dao-Jing X, Ying-Ze Z, Jin W, et al. P38 and ERK1/2 MAPKs act in opposition to regulate BMP9-induced osteogenic differentiation of mesenchymal progenitor cells. BMB Rep. 2012;245(4):247–252.

[35] Cao J, Wei Y, Lian J, et al. Notch signaling pathway promotes osteogenic differentiation of mesenchymal stem cells by enhancing BMP9/Smad signaling[J]. Int J Mol Med. 2017;40:378–388.2865621110.3892/ijmm.2017.3037PMC5504972

